# Clinical Study on the Efficacy of Silver Ion Dressing Combined with Prontosan Gel Dressing in the Treatment of Diabetic Foot Ulcers and the Effect on Serum Inflammatory Factors

This article has been retracted.

**DOI:** 10.1155/2021/2938625

**Published:** 2021-10-23

**Authors:** Da Xu, Tongbin Chu, Guilu Tao

**Affiliations:** ^1^Department of Endocrinology, Zhuji Affiliated Hospital of Shaoxing University, Zhuji, Zhejiang 311800, China; ^2^Department of Wound Repairment, The Second Affiliated Hospital of Dalian Medical University, Dalian, Liaoning 116000, China

## Abstract

Diabetic foot ulcers (DFUs) have a high disability rate and have a great impact on patients and society, and the search for effective and economical treatment options is a major clinical concern. In this study, 112 patients with DFU admitted to two hospitals from October 2018 to November 2020 were randomly divided into 56 cases each in the single group treated with Prontosan gel dressing and the joint group treated on silver ion dressing combined with Prontosan gel dressing. Both groups of patients were evaluated for efficacy after 30 days of treatment. The number of days for debridement, granulation tissue growth time, epithelial tissue formation time, and wound healing time were observed and recorded in both groups. The trauma area, visual analogue score (VAS), and levels of inflammatory factors such as vascular endothelial adhesion molecule-1 (VCAM-1), interleukin-6 (IL-6), tumor necrosis factor-*α* (TNF-*α*), and C-reactive protein (CRP) were recorded before and after treatment in both groups. The occurrence of adverse reactions such as edema, fever, infection, and rash during treatment was recorded in both groups for safety assessment. Comparison of the abovementioned data showed that the clinical efficacy of the joint group was significantly higher than that of the single group. The number of days to clear wounds, granulation tissue growth time, epithelial tissue formation time, and wound healing time were significantly lower in the joint group than in the single group. The trauma area, VAS score, VCAM-1, IL-6, TNF-*α*, and CRP levels decreased in both groups after treatment compared with the pretreatment levels, with the joint group being lower than the single group. The results also showed that the difference in the overall incidence of adverse reactions between the two groups was not statistically significant, and the incidence was low and transient. In addition to the usual treatment regimen of blood glucose control and improvement of microcirculation for patients with DFU, combined treatment with silver ionomer dressings and Prontosan gel dressings can promote ulcer healing and improve foot wound regression. It has a stronger antibacterial effect and can more effectively reduce the inflammatory response of the ulcerated surface with fewer adverse effects, making it an effective and safe method for the treatment of DFU, and has implications for promotion.

## 1. Introduction

Diabetic foot (DF) as one of the serious chronic complications of diabetes mellitus (DM), is the leading cause of hospitalization as well as nontraumatic toe amputation or even amputation in DM patients [1]. Poor long-term glycemic control, diabetic peripheral neuropathy, diabetic peripheral vasculopathy, and local infection may all contribute to the development of DF. Patients with DF who do not receive effective treatment to manage their disease may suffer from reduced skin blood flow, nutritional deficiencies, and decreased body defenses leading to diabetic foot ulcers (DFUs) [2, 3]. In patients with DM, the infection is not easy to clear due to the pathological basis such as poor local blood supply and impaired immune defense function, while the involvement of multiple inflammatory factors leading to systemic inflammation is an important reason that affects the development of DFU into gangrene, osteomyelitis, and even amputation [4]. Therefore, the correct treatment of DFU patients can be of great significance.

Chronic wounds such as DFU are unable to undergo a series of normal and orderly repair processes to achieve anatomical and functional healing within a specified time, which makes the healing cycle prolonged [5]. The traditional concept believes that sufficient oxygen should be given to wound healing and the wound surface should be kept dry, but with the introduction of the “moist healing” philosophy and its continuous practice and confirmation, more and more clinical practitioners are realizing that wounds heal much faster in a wet environment than in a dry one [6, 7]. New dressings developed based on the concept of moist healing have widely replaced traditional dressings. Foam dressings, honey dressings, hydrogel dressings, and silver ion dressings are the most commonly used dressings in clinical wound treatment [8, 9]. Silver ion dressing on the ulcerated surface of diabetic foot can form a local antibacterial environment to reduce the chance of bacterial infection and, thus, reduce local secretion, with bactericidal and antibacterial effects and absorption of wound exudate [10, 11]. Prontosan gel has a long-lasting preventive effect against bacterial biofilm, provides moisture to the wound, and can cause autolysis of necrotic tissue in the DF to promote wound healing [12]. Both dressings are widely used in the treatment of DFU and have good results, but there are relatively few reports on the efficacy of their combined application on DFU.

In this study, the silver ion dressing and Prontosan gel dressing were combined to explore the role of the combination of the two in DFU treatment through clinical research. The clinical data, treatment, and inflammatory factor levels of DFU patients admitted to our hospital were calculated and analyzed, and it was proposed to investigate the clinical effect of silver ion dressing combined with Prontosan gel in the treatment of DFU.

## 2. Case Data and Methods

### 2.1. Case Data

The clinical data of 112 DFU patients admitted from October 2018 to November 2020 were collected. Among them, 71 males and 41 females were aged from 45 to 76 years. All patients were treated with adequate metabolic improvement, nerve nutrition, anti-infection, and wound management after admission to the hospital. After the condition was basically controlled, the patients were randomly divided into a single group receiving Prontosan gel treatment and a joint group receiving silver ion dressing combined with Prontosan gel treatment, with 56 cases each. General data such as age, body mass index (BMI), DM type, duration of DM, duration of DFU, gender, trauma area, blood glucose (BG), Wanger classification, and other DM complications were compared between the two groups, and the differences were not statistically significant (*P* < 0.05, Table 1) and were comparable.

### 2.2. Inclusion Criteria

1. All patients met the relevant diagnostic criteria for DM [13] and had concurrent DFU
2. Patients with foot ulcers of grade II–IV according to the Wanger grading criteria [14]
3. The trauma area was 2 cm^2^∼10 cm^2^
4. Patients were informed about the study and had signed a consent form

### 2.3. Exclusion Criteria

1. Patients with a combination of severe mental or cognitive impairment and noncooperation
2. Foot ulcers caused by diseases such as syphilis, tuberculosis, and cancer
3. Patients with a combination of gangrene, osteomyelitis, severe primary disease of vital organs, and hematologic disorders
4. Women who were pregnant or breastfeeding
5. Patients who were allergic to the local application of silver ionomer dressings and Plantronics gel
6. Patients aged >85 years
7. Patients who had taken hormonal drugs within the last 1 month

### 2.4. Treatment Methods

1. Basic treatment: after admission, all patients were given diabetic diet, active blood glucose control, nerve nutrition, improvement of microcirculation, and other conventional treatments. For patients with more serious foot infection, we chose reasonable antibacterial drugs for systemic anti-infection treatment. According to the specific situation of the wound, different methods of wound cleaning such as peroxide cleaning and negative pressure suction were adopted. After the abovementioned treatment, the patient's blood glucose was well controlled and the local wound bed was well prepared for treatment with additional dressing.
2. Single group: sterile gauze was used to moisten Prontosan liquid gel, and the dressing was covered on the foot trauma and kept for 15 minutes, while the trauma was rinsed with Prontosan liquid gel, and after wiping the trauma clean with sterile cotton swabs, the trauma was well covered by cutting the dressing with suitability according to the trauma characteristics. If the wound is deep and narrow, or even has a sinus tract, filler strips of appropriate size can be placed in it first, filling it as evenly as possible to avoid piling up. The size of the wound was observed, and sterile dry gauze was applied as an outer excipient and fixed by bandages with the right degree of tightness to avoid excessive pressure leading to poor local blood circulation, and the dressing was changed every 24 hours. For the trauma with more exudate and odor, the frequency of dressing change can be enhanced and the dressing can be changed in a timely manner, with every 12 hours being appropriate.
3. Joint group: combined with silver ion dressing on top of Prontosan gel, Prontosan gel was used as in the single group, but silver ion dressing was added on top of the gel to cover the wound immediately after rinsing the wound, and the covering method and replacement frequency are essentially the same as for the single group.

### 2.5. Observation Index

1. The treatment of both groups was observed and compared: the time to debridement, time to granulation tissue growth, time to epithelial formation, and time to wound healing were collected and compared between the two groups. For patients whose wounds had not healed after 30 days of treatment, the original treatment plan was still adopted until the wounds heal, and the patients were followed up and the time of healing is recorded.
2. Trauma area and visual analogue score (VAS) were assessed and compared before and after treatment in both groups: the trauma surface was photographed by the same clinician before treatment, at week 1, week 2, and week 4 of treatment, and the foot ulcer trauma area was measured using image processing software. The VAS score was evaluated before treatment and after 30 d of treatment in all patients by a dedicated person. The side with scales was turned away from the patient when using, and the patient was asked to mark the corresponding location on the straightedge that would represent his or her ability to indicate his or her pain level. The physician gave the patient a score based on the location marked by the patient. The clinical rating was 0 for no pain; 1 to 3 for mild pain but tolerable; 4 to 6 for the patient to have pain and affect sleep, and still tolerable; and 7 to 10 for intense pain, which affects appetite and sleep and is unbearable.

### 2.6. Evaluation of Efficacy

The healing of DFU in both groups was observed before treatment and 30 days after treatment. Cured: the DFU patient's skin color returns to normal, and clinical symptoms disappear completely. Markedly effective: the patient's skin color improved significantly after treatment, the dorsalis pedis artery had rebound force, the wound healing rate was >80%, and the Wagner grading down >2 levels. Valid: clinical symptoms were improved, the dorsalis pedis artery was palpable, skin color of the foot was slightly improved, wound healing rate was 40%∼80%, and the Wagner grade down 1 level. Invalid: no significant improvement in trauma or the need for amputation. Total effective rate = (cured + markedly effective + valid) number of cases/total number of cases × 100%.

### 2.7. Statistical Methods

SPSS 20.0 statistical software was used for statistical analysis of the data, and Prism 8.0 was used for graphing. Clinical efficacy, incidence of adverse reactions, and other count data were expressed as (*n*, %), and a chi-square (*χ*^2^) test was performed. Measures such as mean days to debridement and VAS scores were expressed as mean ± standard deviation (mean ± SD), and a *t*-test was used between the two groups. *P* < 0.05 indicated a statistical difference.

## 3. Results

### 3.1. Comparison of the Clinical Efficacy of the Two Groups

The clinical outcomes of the patients were evaluated and compared after 30 days of treatment. In the single group, 14, 20, 10, and 12 patients were cured, markedly effective, valid, and invalid, respectively, with a total effective rate of 78.57% (44/56). In the joint group, 20, 26, 6, and 4 cases were cured, markedly effective, valid, and invalid, respectively, with a total effective rate of 92.86% (52/56). The total effective rate of the joint group was higher than that of the single group, and the difference was statistically significant (*P* < 0.05, Figure 1).

### 3.2. Comparison of the Indexes between the Two Groups after Treatment

The indexes of the two groups after treatment were observed and recorded. The results showed that the mean days of debridement, days of granulation tissue growth, epithelial tissue formation time, and wound healing time were shorter in the joint group than in the single group, and the difference was statistically significant (*P* > 0.05, Figure 2).

### 3.3. Comparison of Trauma Area and VAS Score before and after Treatment between the Two Groups

The trauma area and VAS score were evaluated before and after treatment. The results showed that there was no statistically significant difference in the trauma area and VAS scores between the two groups before treatment (*P* > 0.05). After treatment, the trauma area and the VAS scores decreased in both groups, with the joint group being lower than the single group, and the difference was statistically significant (*P* < 0.05) (Figure 3).

### 3.4. Comparison of Inflammatory Factor Levels before and after Treatment between the Two Groups

Data such as the levels of inflammatory factors such as VACM-1 before and after 30 days of treatment were collected and compared between the two groups. The results showed that there was no statistically significant difference between the levels of VCAM-1, IL-6, TNF-*α*, CRP, etc. in the two groups before treatment (*P* > 0.05). After treatment, the levels of VCAM-1, IL-6, TNF-*α*, CRP, etc. in both groups were lower than before treatment, and the levels of each factor in the joint group were lower than those in the single group, and the difference was statistically significant (*P* < 0.05) (Figure 4).

### 3.5. Comparison of the Incidence of Adverse Reactions between the Two Groups

The more significant local adverse reactions that occurred during the treatment were counted in both groups. In the single group, there were 2 cases of edema, 1 case of fever, 3 cases of infection, and 2 cases of rash during the treatment period, with a total incidence of local adverse reactions of 14.29% (8/56). In the joint group, there were 3 cases of edema, 1 case of fever, 1 case of infection, and 1 case of rash, with a total incidence of local adverse reactions of 10.71% (6/56). The results showed a statistically significant difference in the total incidence of adverse reactions between the two groups (*P* > 0.05, Figure 5). Local adverse reactions showed a transient nature in both groups.

## 4. Discussion

DF is mostly caused by peripheral neuropathy, peripheral vascularity, and infection. Various types of lesions can cause a lack of protective sensation for pain in the patient's lower limbs, elevated pressure sensory thresholds, muscle atrophy in the lower limbs, and severe toe deformities [15]. If the lesion is not treated promptly and effectively, peripheral vascular lesions may cause local tissue ischaemia and hypoxia in the lower limbs, reducing the immunity of the body and increasing the risk of foot infection [16]. The combination of local infection is a major risk factor for recovery from diabetic foot disease. Local inflammatory response is a protective response to a noxious stimulus, but excessive inflammation can exacerbate the damage, and it has been shown that high levels of inflammatory factors are closely associated with the persistence of DFU [17, 18]. The current treatment of DFU includes glycemic control, improvement of microcirculation, improvement of neurological function, topical dressing of the trauma, and revascularisation [19]. The use of topical dressings on the wound is an important aspect of DFU treatment, and studies have shown that early and effective topical dressings can promote ulcer healing and reduce the incidence of amputation [20]. Based on this, we used an antibacterial silver ionomer dressing combined with Plantronics hydrogel to treat DFU patients with topical dressing changes in order to investigate the effect of this treatment protocol on DFU patients.

The results of the study showed that the overall treatment efficiency of the joint group treated with antibacterial silver ion dressing combined with Prontosan gel was significantly higher than that of the control group treated with Prontosan gel only, and the number of days for debridement, the number of days for granulation tissue growth, and the area of the wound after 30 days of treatment in terms of VAS score were all lower in the joint group than in the single group. This suggests that silver ion dressing combined with Prontosan gel dressing treatment can promote the healing of the patient's ulcer and reduce the patient's pain, which is more effective. Silver ion dressings contain rapidly absorbent and water-locking alginate fibres that draw wound exudate and microorganisms into the dressing and remove them by removing the dressing, reducing impregnation damage to the wound and surrounding skin. Alginate fibres absorb exudate and form a gel, providing a humid microacidic environment to stimulate local vascular proliferation, promote granulation tissue growth, accelerate wound healing, and retain the release of active substances from the exudate, facilitating self-soluble wound debridement [21, 22]. Prontosan gel dressing contains the surfactants undecylenamidopropyl betaine and polihexanide, which are highly compatible with antimicrobial dressings such as silver ions. Also, undecylenamidopropyl betaine significantly enhances the penetration of difficult-to-remove wound coverings with a high ability to remove traumatic tissue debris, bacteria, and biofilms [23]. The use of combination therapy is, therefore, more effective in removing necrotic tissue, preventing biofilm formation, removing exudate in a timely manner, and improving the regression of the foot wound.

VCAM-1, IL-6, and TNF-*α* are all important inflammatory transmitters in DF and mediate the local inflammatory response in DF; CRP is an acute-phase protein that induces the secretion of a variety of inflammatory mediators, including endothelial cells and is positively correlated with the severity of DF infection [24]. The results showed that the levels of VCAM-1, IL-6, TNF-*α*, and CRP in the joint group were significantly lower than those in the single group, suggesting that combination therapy is more advantageous in improving the systemic inflammatory response and clearing serum inflammatory factors in DFU patients. Silver ions have a broad-spectrum antibacterial effect and have a strong inhibitory effect on *Pseudomonas aeruginosa*, *Staphylococcus aureus*, and *Streptococcus* and do not produce drug resistance [25]. Silver ions can bind to enzymes and DNA in the cell walls of protein-organised microorganisms to interfere with bacterial gene replication functions, thus achieving an antibacterial effect, and silver ions can be freed from inactive bacteria to repeat sterilisation with long-lasting effects [26]. Furthermore, the polyhexylguanidine in Prontosan gel also exerts an antibacterial effect by splitting the bacterial cover and dissolving the denatured proteins to prevent and remove the bacterial biofilm, effectively reducing the risk of wound infection [27]. In addition, the incidence of local adverse reactions was low and transient in both groups, suggesting that the combination therapy is an effective and safe treatment for DFU without causing major damage to the body while improving efficacy. Analysing the reasons for this, silver ions as a purely natural broad-spectrum bactericidal agent do not develop drug resistance, the heavy metal components do not volatilise, covering the skin surface does not cause silver toxicity in patients, and has no toxic effect on the body's own cells; the combination therapy is, thus, safe [28].

In addition to the usual treatment regimen of blood glucose control and improvement of microcirculation for patients with DFU, combined treatment with silver ionomer dressings and Prontosan gel dressings can promote ulcer healing and improve foot wound regression. It has a stronger antibacterial effect and can more effectively reduce the inflammatory response of the ulcerated surface with fewer adverse effects, making it an effective and safe method for the treatment of DFU, and has implications for promotion.

## Figures and Tables

**Figure 1:** Comparison of clinical efficacy between the single group and the joint group. Compared with the single group, ^#^*P* < 0.05.

**Figure 2:** Comparison of the indexes between the single group and the joint group after treatment. (a) Average days of debridement. (b) Average granulation tissue growth days. (c) Average epithelial tissue formation time. (d) Average trauma healing time. Compared with the single group, ^#^*P* < 0.05.

**Figure 3:** Comparison of trauma area and VAS scores before and after treatment in the single and joint groups. (a) Average trauma area. (b) Average VAS score. Compared with the same group before treatment, ^*∗*^*P* < 0.05. Compared with the single group of the same period, ^#^*P* < 0.05.

**Figure 4:** Comparison of inflammatory factor levels before and after treatment in the single and joint groups. (a) Average VCAM-1 levels. (b) Average IL-6 levels. (c) Average TNF-*α* levels. (d) Average CRP levels. Compared with the same group before treatment, ^*∗*^*P* < 0.05. Compared with the single group of the same period, ^#^*P* < 0.05.

**Figure 5:** Comparison of the incidence of various adverse reactions and total adverse reactions in the single and joint groups.

**Table 1:** Comparison of basic information between the single group and the joint group.

Information	Single group (*n* = 56)	Joint group (*n* = 56)	*t* or *χ*^2^ value	*P* value
Age (years, mean ± SD)	57.22 ± 9.91	57.41 ± 10.06	0.101	0.920
BMI (kg/m^2^)	23.57 ± 2.69	22.89 ± 2.41	1.409	0.162
*DM typing (n, %)*				
Type 1	2 (3.57)	4 (7.14)	0.704	0.401
Type 2	54 (96.43)	52 (92.86)		

Duration of DM (years, mean ± SD)	10.36 ± 3.16	10.45 ± 3.32	0.147	0.883
Duration of DFU (days, mean ± SD)	57.46 ± 11.46	58.59 ± 12.07	0.508	0.612
*Gender (n, %)*				
Male	34 (60.71)	37 (66.07)	0.346	0.556
Female	22 (39.29)	19 (33.93)		

*DM complications (n, %)*				
Peripheral neuropathy	12 (21.43)	8 (14.29)	0.974	0.324
Ocular complications	7 (12.50)	9 (16.07)	0.292	0.589
Peripheral vascular disease	52 (92.86)	49 (87.50)	0.907	0.341
Nephrotic lesion	45 (80.36)	48 (85.71)	0.571	0.450

Trauma area (cm^2^, mean ± SD)	6.59 ± 0.51	6.73 ± 0.62	1.305	0.195
BG (mmol/L, mean ± SD)	10.41 ± 2.78	10.39 ± 2.64	0.039	0.969
*Wanger grading (n, %)*				
Grade II	22 (39.29)	20 (35.71)	0.805	0.669
Grade III	29 (51.79)	28 (50.00)		
Grade IV	5 (8.93)	8 (14.29)		

## Data Availability

The data during the current study are available from the corresponding author on reasonable request.
